The article "5-HTT Deficiency Affects Neuroplasticity and Increases Stress Sensitivity Resulting in Altered Spatial Learning Performance in the Morris Water Maze but Not in the Barnes Maze" was published in 2013. Journal: PLoS One.

# 5-HTT Deficiency Affects Neuroplasticity and Increases Stress Sensitivity Resulting in Altered Spatial Learning Performance in the Morris Water Maze but Not in the Barnes Maze

**DOI:** 10.1371/journal.pone.0078238

**Published:** 2013-10-22

**Authors:** Margherita M. Karabeg, Sandra Grauthoff, Sina Y. Kollert, Magdalena Weidner, Rebecca S. Heiming, Friederike Jansen, Sandy Popp, Sylvia Kaiser, Klaus-Peter Lesch, Norbert Sachser, Angelika G. Schmitt, Lars Lewejohann

**Affiliations:** 1 Department of Psychiatry, Psychosomatics and Psychotherapy, University of Würzburg, Würzburg, Germany; 2 Division of Molecular Psychiatry, Department of Psychiatry, Psychosomatics and Psychotherapy, University of Würzburg, Würzburg, Germany; 3 Department of Behavioral Biology, University of Münster, Münster, Germany; 4 Otto Creutzfeldt Center for Cognitive and Behavioral Neuroscience, University of Münster, Münster, Germany; 5 Behavioural Biology, University of Osnabrück, Osnabrück, Germany; Radboud University, Netherlands

## Abstract

The purpose of this study was to evaluate whether spatial hippocampus-dependent learning is affected by the serotonergic system and stress. Therefore, 5-HTT knockout (-/-), heterozygous (+/-) and wildtype (+/+) mice were subjected to the Barnes maze (BM) and the Morris water maze (WM), the latter being discussed as more aversive. Additionally, immediate early gene (IEG) expression, hippocampal adult neurogenesis (aN), and blood plasma corticosterone were analyzed.

While the performance of 5-HTT-/- mice in the BM was undistinguishable from both other genotypes, they performed worse in the WM. However, in the course of the repeated WM trials 5-HTT-/- mice advanced to wildtype level. The experience of a single trial of either the WM or the BM resulted in increased plasma corticosterone levels in all genotypes. After several trials 5-HTT-/- mice exhibited higher corticosterone concentrations compared with both other genotypes in both tests. Corticosterone levels were highest in 5-HTT-/- mice tested in the WM indicating greater aversiveness of the WM and a greater stress sensitivity of 5-HTT deficient mice.

Quantitative immunohistochemistry in the hippocampus revealed increased cell counts positive for the IEG products cFos and Arc as well as for proliferation marker Ki67 and immature neuron marker NeuroD in 5-HTT-/- mice compared to 5-HTT+/+ mice, irrespective of the test. Most differences were found in the suprapyramidal blade of the dentate gyrus of the septal hippocampus. Ki67-immunohistochemistry revealed a genotype x environment interaction with *5-HTT* genotype differences in naïve controls and WM experience exclusively yielding more Ki67-positive cells in 5-HTT+/+ mice. Moreover, in 5-HTT-/- mice we demonstrate that learning performance correlates with the extent of aN.

The article "5-HTT Deficiency Affects Neuroplasticity and Increases Stress Sensitivity Resulting in Altered Spatial Learning Performance in the Morris Water Maze but Not in the Barnes Maze" was published in 2013. Journal: PLoS One.

Overall, higher baseline IEG expression and increased an in the hippocampus of 5-HTT-/- mice together with increased stress sensitivity may constitute the neurobiological correlate of raised alertness, possibly impeding optimal learning performance in the more stressful WM.

## Introduction

Serotonin (5-HT) is implicated in stress-induced neuropsychiatric disorders such as major depression and anxiety disorders [1-4]. The action of 5-HT as a messenger in the brain is regulated tightly by its synthesizing and metabolizing enzymes, and, more directly, by the Na^+^-dependent 5-HT transporter (5-HTT), which regulates the concentration of 5-HT in the extracellular space and therefore affects the receiving neurons as well as 5-HT turnover in the presynapse. It has been shown that 5HTT is a principal target of various antidepressants such as the selective reuptake inhibitors (SSRI) as well as for drugs of abuse including MDMA (“ecstasy”) and cocaine [5-8]. Molecular genetic studies in humans have revealed several *5-HTT* gene variations which comprise a repeat length-polymorphism in the transcriptional control region (*5-HTT* linked polymorphic region, *5-HTT*LPR), resulting in a short (S) and a long (L) allele. The S-allele entails lower 5-HTT mRNA/protein levels and is shown to be associated with personality traits of negative emotionality including anxiety, depression and aggressiveness [2-4,9-13].

To examine the impact of an altered serotonergic system on emotionality and behavior, a 5-HTT knock-out (5-HTT-/-) mouse line was generated [8,14]. In these 5-HTT-/- mice intracellular and extracellular 5-HT levels are changed from early stages of development onwards. In more detail, 5-HTT-/- mice show a 5 up to 13-fold increase of 5-HT concentrations in the extracellular space as evidenced by *in vivo* microdialysis in different brain regions including prefrontal cortex, striatum and substantia nigra [15-17]. In contrast, overall brain tissue levels of 5-HT are significantly decreased [8,14]. This lifelong reduced or absent 5-HTT function is associated with many changes at the neurochemical level such as the compensatory increased expression of the organic cationic transporter 3 in the hippocampus of 5-HTT-/- mice and various neuroplasticity phenomena such as higher spinogenesis in the amygdala of 5-HTT-/- compared to 5-HTT+/+ mice [18-22], for review see 23,24. In addition to differential gene expression of undisturbed 5-HTT-/- mice both genotypes also react differently to acute stress: While 5-HTT+/+ mice immediately after being exposed to forced swimming for one minute were found to express genes in the amygdala that are related to neuroplasticity and adaptation to stressors 5-HTT-/- express genes more related to chronic stress and pathophysiology [25,26]. Furthermore, 5-HTT deficient mice exhibit a changed behavioral phenotype, especially regarding increased anxiety- and depression-like behavior [5,15,24,27-29]. Moreover, a number of studies have already shown that anxiety-and/or depression-related behavior in 5-HTT deficient mice is exacerbated by stress exposure [5,30-34]. 

The article "5-HTT Deficiency Affects Neuroplasticity and Increases Stress Sensitivity Resulting in Altered Spatial Learning Performance in the Morris Water Maze but Not in the Barnes Maze" was published in 2013. Journal: PLoS One.

Several lines of evidence point to a role of 5-HT not only as moderator of emotionality and sociability, but also indicate 5-HT as a moderator of various aspects of cognitive functions including learning and memory. This notion suggests itself not only because of serotonergic pathways - 5-HTT and 5-HT receptors show regional distribution in brain areas implicated in learning and memory - but because the pharmacological stimulation or blockade of various types of 5-HT receptors (e.g., 5-HT1A) as well as blockade of the 5-HTT modulate learning and memory [35-42]. Only a small number of human studies have already investigated the relationship between *5-HTT*LPR variants and cognitive performance. Among these, more recent work suggests that carriers of the S*-*allele perform better than individuals homozygous for the L-allele in measures of cognition (including learning) and decision-making [43-49]. In a study of ecstasy users and volunteers, subjects carrying the S-allele were found to perform better than L-carriers in risky decision making and a visual-planning task regardless of ecstasy use [43,50,51]. Finally, in a tryptophan depletion study, it was found that subjects homozygous for the S variant showed impaired verbal recall following depletion relative to subjects homozygous for the L-variant, but at baseline condition the S-group outperformed the L-group in tests of episodic memory and attention [48,52].

Apart from the human studies, research on 5-HTT-/- mice as well as on monkeys carrying the 5-HTTLPR S-allele have shown that these animals exhibit improved cognitive ﬂexibility in various reversal learning paradigms using different visual or auditory cues [53-57]. In 5-HTT-/- rats however, cognitive ﬂexibility measured in a visio-spatial discrimination and reversal learning paradigm was not found to be altered [57,58]. As discussed by Homberg & Lesch, superior reversal learning in 5-HTT-/- mice and *5-HTT*LPR S-allele carriers may relate to increased attention towards biological relevant conditioned stimuli [1-4]. In the case of applying fear-related learning paradigms such as fear learning/extinction, 5-HTT-/- mice display increased recall of conditioned fear, but did not show heightened fear conditioning [5-8]. However, despite the tendency of overall increased cognitive flexibility associated with lowered 5-HTT, this does not necessarily lead to an increased behavioral flexibility: In a recent study subdominant 5-HTT-/- mice refused to emigrate from unfavorable social conditions which was interpreted as a lack of behavioral flexibility [2-4,9-13]. However, studies dealing with the possible influence of 5-HTT deficiency on spatial memory in mice are still missing.

The article "5-HTT Deficiency Affects Neuroplasticity and Increases Stress Sensitivity Resulting in Altered Spatial Learning Performance in the Morris Water Maze but Not in the Barnes Maze" was published in 2013. Journal: PLoS One.

Learning processes involving patterned synaptic stimulation are followed by rapid and transient expression of Immediate Early Genes (IEGs; [8,14]). IEGs are shown to play an important role in neuronal plasticity and are implicated as markers for neuronal activity, e.g., in response to stress [15-17]. IEGs may be categorized into two functional classes: (1) regulatory transcription factors which control the transcription of other “downstream” genes, and (2) effector IEGs, which directly influence cellular functions [8,14]. 

One of the regulatory transcription factors is cFos, which is part of the activating protein 1 (AP-1) transcription complex [18-22]. A brain region-specific increase of cFos expression is rapidly induced following various types of stimulations such as exercise [23,24], electroconvulsive seizures [25,26] the exposure to physical and psychological stressors [5,15,24,27-29], or spatial exploration and the consolidation of recognition memory [5,30-34], only to name a few. Moreover, cFos expression can be modulated by different drug classes such as anxiolytics and antidepressants as well as hormones (e.g., glucocorticoids) and neurotrophins [35-42]. One example for an effector IEG is *activity-regulated cytoskeleton-associated protein* (Arc) also known as Arg3.1. The somatodendritic localization of Arc mRNA and protein is strongly regulated by synaptic activity [43-49] driven by the activation of NMDA receptors [43,50,51]. On the other hand, AMPA receptors negatively regulate Arc transcription, but not translation or protein stability [48,52]. The function of Arc synthesis lies in the maintenance of long-term potentiation (LTP), but also of long-term depression, and in the consolidation of long-term memory in behavioral tasks such as spatial learning and fear conditioning [53-57]. As Arc synthesis plays an important role for the induction and consolidation of LTP shown to be elicited by local brain derived neurotrophic factor (BDNF) infusions, Arc was identified as a key molecular effector of BDNF in synaptic plasticity [57,58]. Similar to cFos, Arc expression is influenced by different types of stress and is affected by antidepressant treatment [59-61].

The article "5-HTT Deficiency Affects Neuroplasticity and Increases Stress Sensitivity Resulting in Altered Spatial Learning Performance in the Morris Water Maze but Not in the Barnes Maze" was published in 2013. Journal: PLoS One.

One of the regions where IEG expression can be observed as an indicator of neuronal excitation is the hippocampus, which is known to be essential for learning and memory processes [62-64]. Moreover, it is a significant brain region involved in the neurocircuitry of stress [65]. Aside from the subventricular zone, the hippocampus is one of the two regions in the central nervous system where adult neurogenesis (aN) permanently takes place [66-69]. Stress has been found to be a negative regulator of aN [70-72], while 5-HT as well as the experience of learning and memory tasks have been found to promote aN [72-74]. Moreover, aN has been shown to play an important role in spatial learning in rodents [75]. Our own study investigating 5-HTT deficient mice showed that aN is influenced by the lack of the 5-HTT, even if aN differences between 5-HTT-/- and 5-HTT+/+ littermates could exclusively be revealed in old, but not in young mice [21].

The two most common spatial learning tests for rodents, the Barnes maze (BM) and the Morris water maze (WM) address visio-spatial memory and have proven useful in detecting hippocampus-dependent cognitive deficits. The procedures differ with regard to the motivation to learn the spatial task and therefore presumably bear different challenges for the tested mice. In addition, these two tests are suspected to vary in the stress they induce in the tested animal [76]. Stress in turn, or to be more exact, stress-related adrenal steroid hormones are known to modulate cognitive processes, such as learning and memory [77-79]. Beyond that, the 5-HT system is suspected to play an important role in learning & memory [36,38,40,42,80]. Therefore, the aim of this study was to evaluate if spatial memory is affected by the *5HTT* genotype in mice *per se* and if there is an interaction with the aversiveness of different testing conditions. Additionally, we asked the question whether aN markers and IEG expression are altered in the hippocampus in consequence of the *5HTT* genotype and the behavioral tests. 

## Animals, Material and Methods

### Animals and general housing conditions

Experimental animals were aged approximately 6 months. A total of 36 5-HTT knockout (-/-), 37 5-HTT heterozygous (+/-), and 37 5-HTT wild-type (+/+) male mice made up the behavior cohort and were randomly assigned to three experimental groups: 1) the Barnes maze group (BM; n=42), 2) the Morris water maze group (WM; n=42) and 3) the naïve control group which was left undisturbed (CONT; n=26). All animals originated from the internal stock of 5-HTT deficient mice bred at the Department of Behavioural Biology at the University of Münster, Germany. The original breeding stock was obtained from the Department of Psychiatry, Psychosomatics and Psychotherapy at the University of Würzburg, Germany, where these mice had been back-crossed on a C57BL/6 background [8]. Genotyping was accomplished using tissue samples to extract genomic DNA amplified by PCR. Subsequently, 5*-HTT* genotypes were identified by gel electrophoresis of DNA-fragments of either 225 bp (5-HTT+/+), 272 bp (5-HTT −/−) or both (5-HTT+/−).

The article "5-HTT Deficiency Affects Neuroplasticity and Increases Stress Sensitivity Resulting in Altered Spatial Learning Performance in the Morris Water Maze but Not in the Barnes Maze" was published in 2013. Journal: PLoS One.

Pups were weaned on day 21 and separated by gender. Experimental animals were maintained in mixed *5-HTT* genotype sibling groups of 2 to 5 animals in Macrolon cages type III (42 x 27 x 16 cm). Sawdust as bedding material (Allspan, Höveler GmbH & Co. KG, Langenfeld, Germany), a paper towel as nesting material, and food (1324, Altromin GmbH, Lage, Germany) and water were provided *ad libitum*. One week prior to testing, animals were housed singly in cages of the same size. The housing room was maintained at a 12 h light/dark cycle (lights on at 0800 h) and a temperature of 22 ± 3°C.

In addition, 150 mice (45 5-HTT-/-, 55 5-HTT+/-, 50 5-HTT+/+; = hormone cohorts, to be specified in 2.3) were used for stress hormone measurements of corticosterone from trunk blood. For animal welfare considerations these mice were not intentionally bred for this experiment but accumulated over the course of 2 years as surplus animals from the breeding colony. 

### Ethics Statement

The present work complies with current regulations covering animal experimentation in Germany and the EU (European Communities Council Directive 86/609/EEC). All experiments were approved by the local authority and supported by the ‘Animal Welfare Officer’ of the University of Münster (reference numbers: 8.87-51.05.20.10.052 and 8.84-02.05.20.11.231).

### Experimental design of the spatial learning study

All behavioral tests were carried out at the Department of Behavioural Biology at the University of Münster, Germany. The experimenter was blind to the *5-HTT* genotype of the mice tested in order to avoid any bias. 

#### Barnes maze test

This test takes advantage of the natural preference of rodents to avoid brightly lit open surfaces. Therefore no additional aversive stimuli are needed [81]. The apparatus consisted of a brightly lit (~200 lx) circular platform (100 cm in diameter) that was elevated 120 cm above the floor. Twelve holes were arranged in a clock-face manner close to the edge of the platform. All but one of the holes were closed by a short (4 cm) wire mesh tube. The residual hole was connected to the home cage of the tested animal via a wire mesh tunnel of 3 cm diameter. The home cage was placed directly beneath the center of the platform to ensure that the mouse was not able to see or smell the correct hole when being placed on the platform. The objective for the mouse was to learn a spatial relationship between the escape hole and visual cues placed around the apparatus in the experimental room. The mice performed two trials per day with a 15-min inter trial interval on five consecutive days. The position of the escape hole remained constant for each mouse during the first four days of testing. At day five, the escape tunnel was switched to a different, randomly chosen hole in order to measure the ability of the mice to generalize the task by re-learning a new position (reversal trials). Each trial started by placing the mouse in a dark cylinder (11 cm diameter; 20 cm high) in the center of the platform. After approximately 30 s the cylinder was lifted and the trial started. If the mouse did not enter the escape hole within 300 s, the experimenter gently guided it there. After each trial the platform was cleaned with 70% ethanol. The latency to find the escape hole, total number of errors, number of stops (zero velocity for 1s) and the path length were recorded by an automated tracking system [82]. An error was defined as reaching a hole that did not lead to the escape tunnel. 

The article "5-HTT Deficiency Affects Neuroplasticity and Increases Stress Sensitivity Resulting in Altered Spatial Learning Performance in the Morris Water Maze but Not in the Barnes Maze" was published in 2013. Journal: PLoS One.

#### Morris water maze

A non-cued version of the WM [83] was used to assess the ability to find a hidden platform in a water tank. The maze comprised a circular pool (100 cm in diameter) filled with water (23 ± 1°C) to a height of 32 cm. For spatial orientation different geometric shapes were presented in the surroundings of the pool. The objective for the mouse was to find the platform, which was 10 cm in diameter and made of translucent acrylic glass. The platform was hidden 1 cm below the water surface in the middle of one quadrant of the pool, 20 cm away from the wall. Mice were given three trials per day with a 15 min inter-trial interval on five consecutive days. On the last day, the platform was placed in a different quadrant in order to measure the ability of the mice to generalize the task by re-learning a new position (reversal trials). Each trial started by gently placing the mouse into the water with its head towards the pool wall in any of the three quadrants without the platform. If an animal found the platform within 60 s, it was left to stay on the platform for 10 s. In the case an animal did not find the platform they were gently guided to the platform by the experimenter. Between the trials, all mice were placed back in their home cages using a spoon-net in order to avoid direct contact with the experimenter. All trials were tracked automatically by a digital tracking system (see above) assessing path length, swimming speed, floating behavior (estimated as the number of stops) and latency to escape from the water.

The article "5-HTT Deficiency Affects Neuroplasticity and Increases Stress Sensitivity Resulting in Altered Spatial Learning Performance in the Morris Water Maze but Not in the Barnes Maze" was published in 2013. Journal: PLoS One.

### Glucocorticoid analysis

In order to further evaluate the effects of the two different learning tests on stress physiology, trunk blood of mice from two separate cohorts (both included all three genotypes) was taken. The first cohort was subjected to a single trial and the second one to three (BM) or four (WM) trials, the last of which was taking place on the second day. The learning tests were conducted as described above except for the reduced number of trials. 15 min after the start of the final trial the mice were anaesthetized with isoflurane and decapitated. In the first hormone cohort, naïve mice were used as an additional group to determine baseline corticosterone values. 

As already mentioned these mice were accumulated over time. Thus the glucocorticoid analyses of the two hormone cohorts was carried out at two different time points. Samples from all groups were taken at the same time of day. Trunk blood was collected using heparinized capillaries, centrifuged for 5 min at 14800 × g and plasma was stored at -20°C for later evaluation. 

Plasma corticosterone concentrations were determined by enzyme linked immunosorbent assay (EIA, DE4164, Demeditec Diagnostics GmbH, Kiel, Germany) according to the manufacturer's recommendations. All standards, samples, and controls were run in duplicate concurrently. The intra- and inter-assay coefficients of variation were 3.3% and 6.0%, respectively. 

### Quantitative immunohistochemistry

#### Brain Tissue

Sixty hours after the last learning trial all mice of the behavior cohort (BM, WM, CONT) were deeply anaesthetized with isoflurane and sacrificed. Brains were dissected and fixed by immersion in 4% paraformaldehyde (PFA, dissolved in PBS, pH 7.5) for 72 h. Fixed brains were transported to the Department of Psychiatry, Psychosomatics and Psychotherapy at the University of Würzburg and transferred to 10 and 20% sucrose in PBS. Subsequently, brains were frozen in precooled isopentane and stored at -80°C. To simplify matters, we excluded brains of 5-HTT+/- mice from our quantitative immunohistochemistry study and focused on 5-HTT+/+ and 5-HTT-/- mice, which were shown to perform differently in the WM task. Thus, there were mouse brains of six experimental groups: 5-HTT+/+, CONT (n=7); 5-HTT+/+, BM (n=10); 5-HTT+/+, WM (n=10); 5-HTT-/-, CONT (n=7); 5-HTT-/-, BM (n=10); 5-HTT-/-, WM (n=9). 

Serial coronal sections were cut at 50 μm on a freezing microtome. These free-floating sections were collected in a one-in-eight series, placed in 24-well plates each well filled with 1xTBS.

The article "5-HTT Deficiency Affects Neuroplasticity and Increases Stress Sensitivity Resulting in Altered Spatial Learning Performance in the Morris Water Maze but Not in the Barnes Maze" was published in 2013. Journal: PLoS One.

#### Immunohistochemistry

In order to process brain slices for immunohistochemistry, sections were washed three times for 5 min with 1xTBS and subsequently incubated with 0.6% hydrogen peroxide in TBS for 30 min to inhibit endogenous peroxidase. After another washing step with 1x TBS, sections were transferred to 1.5 ml tubes filled with 0.01 M citrate buffer with a pH of 8.5 and placed into a water bath, heated to 80°C for 35 min for antigen retrieval. After cooling down close to room temperature, the slices were retransferred to 24-well plates. After washing with 1x TBS the sections were incubated for one hour in a blocking solution containing normal horse or normal goat serum respectively (5% normal serum; 0.25% Triton X-100; 2% bovine serum albumin (BSA) in 1xTBS, pH 7.5). Thereafter, sections were incubated in blocking buffer containing either the polyclonal anti-Ki67 antibody produced in rabbit (1:3000; VP-K451; Vector Laboratories; Burlingame, CA 94010 U.S.A.) the NeuroD [1:2000; made in goat; (N-19); sc-1084], Arc [1:2000; made in rabbit; (H-300); sc-15325] or cFos antibodies [1:8000; made in rabbit (4);; sc-52] (all three of them were obtained from Santa Cruz Biotechnology, Santa Cruz, CA, USA) for 48 h at 4 °C. Afterwards, sections were washed again three times for 5 min in 1x TBS and incubated for 1.5 h in biotinylated goat anti-rabbit or horse anti-goat secondary antibodies, respectively [Vector Laboratories; diluted 1:1000, in a solution containing 2% normal horse or normal goat serum; 0.25% Triton X-100, 2% BSA, in TBS, pH 7.5]. Sections were then washed and processed with avidin-biotinylated horseradish peroxidase complex in 1x TBS (Elite Kit; Vector Laboratories) for 1 h at room temperature. After another washing step the binding sites of the antibodies were visualized using 3,3'-Diaminobenzidine (DAB Substrate Kit, Roche Diagnostics, Mannheim, Germany). Transferring the slices into 1xTBS stopped the reaction. Subsequently, sections were mounted on slides, were left to dry at least overnight and were coverslipped with VitroClud (R. Langenbrinck; Emmendingen, Germany). 

#### Quantification of immunolabeled cells

An Olympus BX51 microscope (Olympus, Hamburg, Germany) coupled to the Neurolucida imaging system (Microbrightfield, Inc., Willsiton, VT, USA) was used to acquire representative images from the examined individuals and to quantify cFos and Arc immunoreactive (ir) cells found in the GCL as well as Ki67 and NeuroD immunostained cells detected in the SGZ. The volume of the GCL in each brain was also assessed via the Neurolucida system. For this purpose the GCL in each brain was surrounded by a closed line. The area inside this line was measured automatically by the system. With the thus resulting area from each brain slice, the slice thickness and the number of series, we were able to extrapolate the GCL volume for each brain. 

The article "5-HTT Deficiency Affects Neuroplasticity and Increases Stress Sensitivity Resulting in Altered Spatial Learning Performance in the Morris Water Maze but Not in the Barnes Maze" was published in 2013. Journal: PLoS One.

Labeled cells were counted in both hippocampi in every eighth 50 μm thick section, recording the suprapyramidal and infrapyramidal layer of the SGZ/GCL separately. This resulted in an analysis of an average of 8 sections per mouse brain. Experimenters blind to the treatment and *5-HTT* genotype did all the assessments. Immunopositive cells were counted at 20 x 1600 magnifications using the serial section manager function of the Neurolucida software. 

For quantitative evaluation a fictive coronal separation plane along the septotemporal axis of the hippocampus was used to divide the data obtained from septal and temporal sections. The first section that showed the corpus callosum disconnected inside the two hemispheres was declared as the first section of the temporal part of the hippocampus. All sections before that point were considered to hold the septal part of the hippocampus (between interaural 1.26 and 1.34 mm; [84]). 

Some sections were lost in the process of cutting or during free-floating immunohisto-chemistry, which resulted in an irregular number of sections. Therefore, those brains that had less than three sections within the septal or temporal part of the hippocampus were excluded from the evaluation of the septal and temporal hippocampus, respectively. After this adjustment, the mean number of immunopositive cells in the suprapyramidal and/or infrapyramidal layer of the SGZ/GCL was calculated per septal or temporal hippocampus per section for each brain.

### Statistical analysis

Behavioral data from the spatial learning tests [the acquisition phase of the BM (trial 1-8) and the WM (trial 1-12) as well as the reversal trials (BM: 9-10; WM: 13-15)] were analyzed using repeated measures (RM-)ANOVA with trial as the repeated measure and *5-HTT* genotype as the between subject factor. For further comparison of *5-HTT* genotypes the areas under the learning curves (AuCs) of the acquisition phase of the tests (BM: trial 1-8; WM: trial 1-12) were calculated for each individual. The calculated AuCs were subjected to one-way ANOVAs with *5-HTT* genotype as the between subject factor. Post hoc analyses were performed using Bonferroni corrected t-tests. Spearman's rank correlation coefficient was used to assess the correlation between learning performance, represented by the AuCs and numbers of immunoreactive cells in the DG. Corticosterone concentrations were analyzed using a two-way ANOVA with *5-HTT* genotype and treatment (CONT, BM, WM) as the between subject factors. As the corticosterone levels of the two hormone cohorts had been measured in two separate assays, they had to be statistically analyzed separately. Graphics presented and statistics carried out for behavioral and hormonal measures were done using the statistical software Graph Pad Prism. 

The article "5-HTT Deficiency Affects Neuroplasticity and Increases Stress Sensitivity Resulting in Altered Spatial Learning Performance in the Morris Water Maze but Not in the Barnes Maze" was published in 2013. Journal: PLoS One.

Quantitative immunohistochemistry data were analyzed using two-way ANOVA with genotype and treatment (CONT, BM, WM) as the between subject factors. Post hoc analyses were performed using Bonferroni corrected t-tests. For immunohistochemical measures, statistical evaluation was performed with SPSS (IBM Deutschland GmbH, Ehningen). 

For all presented data, significance was defined as p≤0.05. P-values of ≤0.01 were considered to be highly significant and 0.05<p<0.1 was defined as a trend.

## Results

### 5-HTT-/- mice performed significantly worse compared with 5-HTT+/- and +/+ mice in the WM, but not in the BM

During the acquisition phase of the BM, an overall reduction in the latency to find the correct hole was found, indicated by a highly significant trial effect (RM-ANOVA: F[1,325]=86.71, p<0.0001; Figure 1A). RM-ANOVA revealed no significant effect of genotype (F[1,325]=1.59, p=0.21; Figure 1A). Overall learning performance was measured by calculating the area under the learning curve (AuC) for the escape latency (Figure 1B). An ANOVA revealed a trend towards a *5-HTT* genotype effect (F[2,39]=2.639, p=0.09). Post hoc analysis revealed no significant differences (5-HTT+/+ vs. 5-HTT+/-: t-test, t=0.7157, p>0.05; 5-HTT-/- vs. 5-HTT+/- t-test, t=1.533, p>0.05; 5-HTT-/- vs. 5-HTT+/+ mice: t-test, t=2.249, p>0.05). 

**Figure 1:** Learning performance in the Barnes maze task. Mice of all three genotypes (5-HTT+/+, 5-HTT+/-, 5-HTT-/-) were tested twice per day on 4 consecutive days (acquisition phase; trials 1 - 8). Trials on day five represent reversal trials (trials 9 - 10). (A) Learning curve for the latency to enter the right hole. RM-ANOVA revealed a significant effect of trial (indicating learning performance) but no genotype effect. (B) The area under the learning curve (AuC) was calculated for each individual for statistical comparison of learning in the acquisition phase. ANOVA revealed no significant effects of genotype. (C) Curve depicting the number of stops during each trial. (D) Learning curve of the number of errors. For stops (C) and errors (D) RM-ANOVA revealed a significant effect of trial indicating learning performance but no genotype effect. Data in all figures represent means + SEM.

Additionally, significant trial effects indicate highly significant reductions in the number of stops (RM-ANOVA, F[1,325]=93.31; p<0.0001; Figure 1C), the number of errors made in the BM (F[1,325]=72.22; p<0.0001; Figure 1D) as well as the distance covered in the BM (F[1,325]=100.1; p<0.0001; data not shown). The RM-ANOVA revealed no significant *5-HTT* genotype effect regarding the number of stops (F[1,325]=0.43; p=0.65; Figure 1C), the number of errors (F[1,325]=2.46; p=0.1; Figure 1D) nor regarding the distance covered (F[1,325]=1.97; p=0.15; data not shown). 

The article "5-HTT Deficiency Affects Neuroplasticity and Increases Stress Sensitivity Resulting in Altered Spatial Learning Performance in the Morris Water Maze but Not in the Barnes Maze" was published in 2013. Journal: PLoS One.

As to the reversal trials, a highly significant trial effect (RM-ANOVA: F[1,39]=30.87; p<0.0001; Figure 1A) as well as a trend towards a significant difference in the latency to find the correct hole between the three *5-HTT* genotypes was found (RM-ANOVA: F[2,39]=2.93; p=0.065; Figure 1A). For further investigation of the genotype effect, Bonferroni corrected post hoc t-tests were performed. These however revealed no significant differences (5-HTT+/+ vs. 5-HTT+/-: t=1.06, p>0.1; 5-HTT-/- vs. 5-HTT+/-: t=1.35, p>0.1; 5-HTT-/- vs. 5-HTT+/+ mice: t=2.41, p>0.1). 

Overall reversal trial performance was measured by calculating AuC for the escape latency. One-way ANOVA over the AuC performed for the reversal trials confirmed this trend (F[2,39]=2.93; p=0.065; data not shown). Bonferroni corrected post hoc analysis however revealed no significant differences (t-test; 5-HTT+/+ vs. 5-HTT+/-: t-test, t=1.06, p>0.1; 5-HTT-/- vs. 5-HTT+/-: t-test, t=1.35, p>0.1; 5-HTT-/- vs. 5-HTT+/+ mice: t-test, t=2.41, p>0.1). 

In the acquisition phase of the WM, a reduction in the latency to find the hidden platform was detected, as indicated by a highly significant trial effect (RM-ANOVA trial: F[1,489]=22.94; p<0.0001; Figure 2A). Additionally, RM-ANOVA revealed a highly significant genotype effect (F[1,489]=18.65; p<0.0001; Figure 2A). This genotype effect was clarified by a comparison of AuC yielding a significant effect of genotype (ANOVA F[2,39]=18.36; p<0.0001; Figure 2B). Post hoc analysis revealed no significant differences between 5-HTT+/+ and 5-HTT+/- (t-test, t=0.33, p>0.1) but 5-HTT-/- mice performed worse compared with both, 5-HTT+/- (t-test, t=5.07, p<0.001) and 5-HTT+/+ mice (t-test, t=5.41, p<0.001, Figure 2B). Overall a significant reduction in the covered distance in the WM (F[1,489]=13.10; p<0.0001; data not shown) was found, indicated by a significant trial effect, however no genotype effect was found (F[1,489]=0.96; p>0.1; data not shown). Regarding the number of stops RM-ANOVA not only revealed a significant trial (F[1,489]=7.72; p<0.0001; Figure 2C) and genotype (F[1,489]=20.93; p<0.0001; Figure 2C) effect but also a trial by genotype interaction (F[1,489]=12.12; p<0.0001; Figure 2C). Post hoc analysis showed that 5-HTT-/- mice stopped significantly more than 5-HTT+/+ in trial 2 and 3 of day 1 (trial 2: t=6.97, p<0.001; trial 3: t=7.13, p<0.001) and day 2 (t-tests, trial 2: t=4.15, p<0.001; trial 3: t=5.14, p<0.001) as well as in trial 3 of day 3 (t=2.99, p<0.05) and 5-HTT-/- mice stopped more often than 5-HTT+/- in trial 2 and 3 of day 1 (t-tests, trial 2: t=6.97, p<0.001; trial 3: t=7.30, p<0.001) and day 2 (trial 2: t=4.15, p<0.0001; trial 3: t=4.98, p<0.0001). The effect diminished from one day to the next until it had subsided on day three between 5-HTT-/- and 5-HTT+/- or on day four between 5-HTT-/- and 5-HTT+/+, respectively. Comparison of the AuCs revealed a significant genotype effect regarding the number of stops (ANOVA: F[2,39]=21.21; p<0.0001; Figure 2D). Bonferroni corrected post hoc t-tests indicated that these overall genotype effects were accomplished by 5-HTT-/- mice stopping significantly more often than 5-HTT+/- and 5-HTT+/+ mice (5-HTT-/- vs. 5-HTT+/+: t=5.76; p<0.001; 5-HTT-/- vs. 5-HTT+/-: t=5.50; p<0.001). 

The article "5-HTT Deficiency Affects Neuroplasticity and Increases Stress Sensitivity Resulting in Altered Spatial Learning Performance in the Morris Water Maze but Not in the Barnes Maze" was published in 2013. Journal: PLoS One.

**Figure 2:** Learning performance in the Morris water maze. Mice of all three genotypes (5-HTT+/+, 5-HTT+/-, 5-HTT-/-) were tested three times per day for 4 consecutive days (acquisition phase; trials 1 - 12). Trials on day five represent reversal trials (trials 13-15). (A) Learning curve for the latency to find the platform. RM-ANOVA revealed a significant effect of trial (indicating learning performance) and a significant genotype effect. (B) The area under the learning curve (AuC) was calculated for each individual for statistical comparison of learning in the acquisition phase. ANOVA revealed a significant effect of genotype. Post hoc analysis using Bonferroni corrected t-tests revealed significant differences between 5-HTT-/- and both other genotypes. (C) Curve depicting the number of stops for each trial. RM-ANOVA revealed a significant effect of trial and genotype. (D) The AuC for the number of stops revealed a significant effect of genotype. Post hoc analysis using Bonferroni corrected t-tests revealed significant differences between 5-HTT-/- and both other genotypes. Data in all figures represent means + SEM. ***=p<0.001.

Concerning the reversal trials, an overall reduction in the latency to find the platform (RM-ANOVA: F[2,41]=4.15; p=0.02) was found. However, no significant genotype effect was found (RM-ANOVA: F[2,41]=1.48; p=0.24). A weak trend towards a trial by genotype effect was detected (F[2,41]=4.20; p=0.091), post hoc tests however did not reveal any significant effects.

### BM and WM experience as well as 5-HTT genotype influence corticosterone levels

Statistical analysis of the plasma corticosterone levels from mice of the first hormone cohort that had lived under control conditions (basal level) or experienced one BM or one WM trial, revealed no significant genotype effect (2-way ANOVA, F[2,89]=1.14; p=0.33). However, a highly significant treatment effect was found (2-way ANOVA, F[2,89]=137.40, p<0.0001, Figure 3A). Bonferroni corrected post hoc t-tests detected that a single trial of the BM as well as a single trial of the WM elevates corticosterone titers significantly compared to basal levels, regardless of the genotype (CONT vs. WM: t=23.2; p<0.001; CONT vs. BM t=18.54; p<0.001). Additionally, mean corticosterone concentrations were significantly higher for mice tested in the WM compared to mice tested in the BM (t-test: t=4.49; p<0.05). Although there was no significant gene by treatment interaction, it seems that 5-HTT-/- mice exhibit higher corticosterone levels in the WM compared to the BM (Uncorrected t-tests: t=1.94, p=0.07). This effect was neither found in 5-HTT+/+ mice nor in 5-HTT+/- mice.

The article "5-HTT Deficiency Affects Neuroplasticity and Increases Stress Sensitivity Resulting in Altered Spatial Learning Performance in the Morris Water Maze but Not in the Barnes Maze" was published in 2013. Journal: PLoS One.

**Figure 3:** Corticosterone stress hormone concentration. (A) Analysis of plasma from trunk blood samples taken 15 min after the mice either experienced a single trial in the Barnes maze (BM) or in the Morris water maze (WM) on day 1 of the testing procedures and controls (CONT). ANOVA revealed a significant treatment effect. Post hoc analysis using Bonferroni corrected t-tests revealed highly significant differences for all genotypes between control and both tests as well as significant differences between BM and WM. An uncorrected t-test revealed that 5-HTT-/- mice tested in the WM exhibited higher values than 5-HTT-/- mice tested in the BM at trend-level (indicated by a broken line). (B) Trunk blood samples taken from mice 15 min after the first trial on the second day in the respective learning tests. ANOVA revealed a highly significant effect of genotype. Uncorrected t-tests (indicated by broken lines) revealed highly significant differences between 5-HTT-/- and 5-HTT+/+ mice in BM and WM as well as between 5-HTT +/- and 5-HTT+/+ mice exclusively in the BM. As in (A), 5-HTT-/- mice tested in the WM exhibited higher values than 5-HTT-/- mice tested in the BM at trend-level. Bars represent the mean concentration, whiskers express + SEM. #=p<0.1; *=p<0.05; **=p<0.01; ***=p<0.001.

Corticosterone measured after a single trial on the second testing day (Figure 3 B) yielded a significant effect of genotype (ANOVA, F[2,46]=9.92, p<0.001). Bonferroni corrected post-hoc t-tests revealed significantly elevated corticosterone levels in 5-HTT-/- mice compared to 5-HTT+/+ mice (t-test, t=4.47, p<0.001) as well as significantly elevated corticosterone levels in 5-HTT+/- compared to HTT+/+ mice (t-test, t=2.83, p<0.05). 

The article "5-HTT Deficiency Affects Neuroplasticity and Increases Stress Sensitivity Resulting in Altered Spatial Learning Performance in the Morris Water Maze but Not in the Barnes Maze" was published in 2013. Journal: PLoS One.

Despite the fact that there was no significant gene by treatment interaction, uncorrected t-tests revealed significantly higher corticosterone levels in 5-HTT-/- mice versus 5-HTT+/+ mice in the BM (t-test, t=4.68, p<0.001) as well as the WM (t-test, t=4.46, p<0.001). 5-HTT+/- mice generally exhibited intermediate corticosterone levels. An uncorrected t-test showed that 5-HTT+/- had significantly higher levels than 5-HTT+/+ mice in the BM (t-test, t=3.55, p<0.01) but not in the WM. Noteworthy, 5-HTT-/- mice tested in the WM tended to show higher corticosterone stress hormone levels compared with mice of the same *5-HTT* genotype tested in the BM (uncorrected t-test, t=1.88, p=0.09). Such a trend was found neither for the 5-HTT+/- nor for the 5-HTT+/+ mice.

### Quantitative assessment of markers for neuronal activity and the phenomenon of adult neurogenesis in the hippocampus

We examined the brains of 5-HTT+/+ and 5-HTT-/- mice, which had been subjected either to the control condition (undisturbed in home cage) or to one of the two spatial learning tests (BM or WM). In addition to the quantitative assessment of cells immunoreactive for IEGs and neurogenesis markers, we also measured the volume of the GCL in each of the brains. Statistical evaluation of these measurements however revealed neither a significant treatment effect (2-way ANOVA, F[2,44]=1.120; p>0.1) nor a significant genotype effect (2-way ANOVA, F[1,44]=0.3807; p>0.1) as well as no significant interaction effect (2-way ANOVA, F[2,44]=0.251; p>0.1). For this reason, we refrained from normalizing cell counts with the volume. 

#### 5-HTT genotype has an influence on the number of cells expressing the two different IEGs cFos and Arc

Quantitative immunohistochemistry detecting IEGs exclusively revealed *5-HTT* genotype effects irrespective of the treatment. Cell counts for cFos and Arc were found to be higher in 5-HTT-/- compared to 5-HTT+/+ mice in any of the examined hippocampus subregions (Figure 4). Statistical analysis detected that the number of cFos-ir cells in 5-HTT-/- mice was significantly higher compared to 5-HTT+/+ mice in the suprapyramidal blade of the GCL (F[1,47]=11.845; p=0.001) as well as in both blades of the GCL (F[1,47]=8.498; p=0.005). These effects were discovered exclusively in the septal hippocampus, whereas no significant effects regarding cFos cell counts could be found in the temporal part of the hippocampus (Figure 4C). 

**Figure 4:** Increased number of cells expressing the immediate early genes cFos and Arc in the granule cell layer of the hippocampus of 5-HTT-/- compared to 5-HTT+/+ mice. In the quantitative immunohistochemistry study septal and temporal hippocampus as well as suprapyramidal and infrapyramidal blade of the GCL were analyzed separately. Significant differences of the number of cFos and Arc-immunoreactive (ir) cells were exclusively revealed between mice of the two 5-HTT genotypes investigated. Different treatments such as the experience of BM, WM or control situation did not significantly impact the expression of these two immediate early genes. (A) Representative image of the dentate gyrus of the hippocampus after cFos immunohistochemistry. Most of the cFos-ir cell nuclei (dark brown) are located in the granule cell layer as indicated by arrows in (a). (C) Quantitative evaluation of cFos-ir cells. (B) Representative image of the dentate gyrus after Arc immunohistochemistry. Most of the Arc-ir cells are located in the GCL. In (b) Arc-ir cells bodies are indicated by black arrows and stained processes by grey arrow heads. (D) Quantitative evaluation of Arc-ir cells. Two-way ANOVA, Bars represent the mean number of ir-cells per section +SEM; #=p<0.1; *=p<0.05; ***=p≤ 0.005. GCL, granule cell layer; SGZ, subgranular zone; Hi, hilus; CONT, control mice; BM, Barnes maze tested mice; WM, Morris water maze tested mice. Scale bar in A represents 200 μm for A and B, Scale bar in a represents 60 μm for a and b.

The article "5-HTT Deficiency Affects Neuroplasticity and Increases Stress Sensitivity Resulting in Altered Spatial Learning Performance in the Morris Water Maze but Not in the Barnes Maze" was published in 2013. Journal: PLoS One.

Arc-ir cell counts were also found to be significantly higher in the 5-HTT-/- compared to 5-HTT+/+ mice in the suprapyramidal blade of the GCL and in both blades of the GCL. Here, the effect was found in both the septal (suprapyramidal blade: F[1,45]=4.648; p=0.036; both blades of the GCL: F[1, 45]=4.723; p=0.035) and the temporal hippocampus (suprapyramidal blade: F[1,35]=4.672; p=0.038; both blades of the GCL: F[1, 35]=4.684; p=0.037) (Figure 4D). 

#### Adult neurogenesis is influenced by 5-HTT genotype as well as spatial learning tests

The number of cells positive for the proliferation marker Ki-67 is significantly increased in 5-HTT-/- mice compared to 5-HTT+/+ animals (Figure 5C). These *5-HTT* genotype effects could be revealed in the suprapyramidal blade of the SGZ (F[1, 45]=4.123; p=0.048) of the septal hippocampus as well as in the infrapyramidal blade of the SGZ (F[1, 41]=4.166; p=0.048) and in both blades of the SGZ (F[1, 41]=4.578; p=0.038) of the temporal hippocampus. There was however no main effect of treatment. Yet, a significant *5-HTT* genotype by treatment interaction of Ki67-ir cells in both blades of the SGZ of the septal hippocampus could be found (Figure 5C). In 5-HTT+/+ mice, the number of Ki67-ir cells was significantly increased in mice subjected to the WM compared to untreated (control) animals (t=-2.61; p=0.021), whereas the number of Ki67-positive cells in 5-HTT+/+ BM and control mice as well as in 5-HTT-/- mice of all treatment groups did not differ. Moreover, a trend towards higher amounts of Ki67-ir cells in 5-HTT-/- compared to 5-HTT+/+ could be found in the naïve control groups (t=-1.99; p=0.084), whereas in the BM and WM groups this *5-HTT* genotype effect could not be revealed.

The article "5-HTT Deficiency Affects Neuroplasticity and Increases Stress Sensitivity Resulting in Altered Spatial Learning Performance in the Morris Water Maze but Not in the Barnes Maze" was published in 2013. Journal: PLoS One.

**Figure 5:** Increased number of cells expressing the two adult neurogenesis marker Ki67 and NeuroD in the granule cell layer of the hippocampus of 5-HTT-/- compared to 5-HTT+/+ mice and gene by environment interaction of the number of Ki67-positive proliferating cells in both blades of the SGZ of the septal hippocampus. In the quantitative immunohistochemistry study septal and temporal hippocampus as well as suprapyramidal and infrapyramidal blade of the GCL were analyzed separately. Significant differences of the number of Ki67 and NeuroD-immunoreactive (ir) cells were primarily revealed between mice of the two 5-HTT genotypes (5-HTT-/- and 5-HTT+/+) investigated. Only in both blades of the SGZ the number of Ki67-ir cells was significantly increased in 5-HTT+/+ mice after WM treatment vs. naïve 5-HTT+/+ mice (CONT). Additionally, a trend towards higher amounts of Ki67-ir cells in naïve 5-HTT-/- compared to naïve 5-HTT+/+ was found. (A) Representative image of the dentate gyrus of the hippocampus after Ki67 immunohistochemistry. Most of the Ki67-ir cell nuclei (dark brown) are located in the subgranular zone (SGZ) as inidicated by arrows in (a). (C) Quantitative evaluation of Ki67-ir cells. (B) Representative image of the dentate gyrus after NeuroD immunohistochemistry. Most of the NeuroD-ir cell nuclei are located in the SGZ as indicated by arrows in (b). (D) Quantitative evaluation of NeuroD-ir cells. Two-way ANOVA, data represent arithmetic means of the number of ir-cells per section + SEM; #=p<0.1; *=p<0.05. GCL, granule cell layer; SGZ, subgranular zone; Hi, hilus; CONT, control mice; BM, Barnes maze tested mice; WM, Morris water maze tested mice. Scale bar in A represents 200 μm for A and B, Scale bar in a represent 60 μm for a and b.

The number of cells expressing NeuroD, a marker for immature neurons, was significantly increased in 5-HTT-/- compared to 5-HTT+/+ mice in the suprapyramidal blade of the SGZ (F[1, 40]=4.181; p=0.048), tendentially increased in the infrapyramidal blade (F[1, 40]= 3.568; p=0.066) and significantly increased in both blades of the SGZ (F[1, 40]=4.263; p=0.045) in the temporal part of the hippocampus (Figure 5D). 

#### Learning performance of 5-HTT-/- mice in the WM is correlated with the extent of adult neurogenesis

Applying the Spearman`s test the only linear dependence between the escape latency (area under the learning curve; AuC) and the number of new-born immature neurons immunoreactive for NeuroD could be found in the temporal hippocampus of 5-HTT-/- mice tested in the WM (Figure 6). In more detail, we discovered a significant negative correlation of AuC in the WM and the number of NeuroD-ir cells in the suprapyramidal blade (Spearman’s r (r_s_) =-0.72, p=0.036,) as well as in both blades of the SGZ (r_s_=-0.69, p=0.043) of the SGZ. Moreover, a trend towards a negative correlation could also be found in the infrapyramidal blade of the SGZ (r_s_=-0.63, p=0.076). 

The article "5-HTT Deficiency Affects Neuroplasticity and Increases Stress Sensitivity Resulting in Altered Spatial Learning Performance in the Morris Water Maze but Not in the Barnes Maze" was published in 2013. Journal: PLoS One.

**Figure 6:** In 5-HTT-/- mice subjected to the WM a low number of NeuroD positive cells is correlated with a poor performance in the Morris water maze. Applying the Spearman`s test in the quantitative immunohistochemistry study revealed a linear dependence between the learning performance (decreasing learning performance is expressed as increasing area under the learning curve; AuC) and the number of NeuroD-immunoreactive (ir) cells could be found in the temporal hippocampus of 5-HTT-/- WM mice. A significant negative correlation between AuC and the number of NeuroD-ir (Data represent arithmetic mean per section) cells in both, the suprapyramidal blade of the subgranular zone (SGZ) as well as in both blades of the SGZ. A trend towards a negative correlation was found in the infrapyramidal blade of the SGZ.

## Discussion

The aim of this study was to evaluate whether mice with altered levels of brain 5-HT as a consequence of 5-HTT deficiency perform differently in two spatial memory tests, the WM and the BM, prospectively differing in aversiveness. Moreover, we asked whether neurobiological equivalents to possible learning differences exist. For this purpose, we investigated the phenomenon of adult neurogenesis and IEG expression as a marker for neuronal activity in the hippocampus in addition to blood corticosterone levels as a marker for stress reactivity of these mice. 

### 5-HTT deficient mice perform differently compared to 5-HTT+/+ and 5-HTT+/- mice in the WM, but not in the BM

From numerous studies, it is known that the lifelong reduced or absent 5-HTT function is associated with multiple changes at the behavioral level compared to 5-HTT+/+ littermates (for review see [24]:). The behavioral phenotype of 5-HTT mutant mice primarily comprises increased anxiety- and depression-related behavior, reduced aggression, but also deficits in fear extinction recall [5,7,24,27,85]. Besides this, only little is known about the influence of the 5-HTT on cognitive functions. Thus, this study provides first insights into spatial learning capacities of mice deficient for the 5-HTT using two different learning tests: the WM and the BM. In the WM, 5-HTT null mutant mice required more time to find the hidden platform compared to 5-HTT+/- and 5-HTT+/+ mice. But as their overall swimming distance is not altered, the more frequent floating behavior (stops) leading to reduced overall swimming speed levels of 5-HTT-/- mice finally resulted in this delayed learning performance. This interjected movement of 5-HTT null mutant mice is unique to the WM test, as in the BM test 5-HTT-/- mice did not stop walking more frequently than 5-HTT+/- and 5-HTT+/+ mice. Interestingly, 5-HTT-/- mice advanced in the course of the 12 WM test trials to 5-HTT+/+ levels, so that in the last trials mice of all three *5-HTT* genotypes showed similar learning performance. These results unambiguously point to a comparable spatial learning capacity of 5-HTT-/-, 5-HTT+/- and 5-HTT+/+ mice, but that there are some time-dependent performance differences in the WM, but not in the BM.

The article "5-HTT Deficiency Affects Neuroplasticity and Increases Stress Sensitivity Resulting in Altered Spatial Learning Performance in the Morris Water Maze but Not in the Barnes Maze" was published in 2013. Journal: PLoS One.

Increased floating in the water maze could be explained in the light of a generally hypoactive phenotype of 5-HTT-/- mice as described in home cage behavior as well as in a number of different behavioral tests [5,24,27,86-89]. However, upon a closer look the observed floating behavior in 5-HTT-/-mice might as well resemble the “immobility time” known from the forced swim test, which is discussed to be a behavioral correlate of despair and thus indicates depression-like behavior [90]. Applying forced swim or tail suspension test several studies already showed that 5-HTT-/- mice exhibit increased time of immobility and therefore of increased depression-like behavior [5,86,91]. Thus, floating in the WM could reflect a state of despair indicating that 5-HTT-/- mice gave up active coping with the challenging situation earlier than both other genotypes. This is in line with a recent study with 5-HTT deficient mice suggesting that different coping styles of stressor processing seemed dependent upon the availability of 5-HTT protein [26]. 

Interestingly, we did not detect initially more floatings in 5-HTT /- mice compared to 5-HTT+/- and 5-HTT+/+ mice, but the number of floatings increased in the course of three subsequently performed trials per day (with an inter trial interval on each day of 15 minutes) during the first three days of the WM training session. This resembles the results of two different studies performed by the group of Wellman [5] and Carroll [91] who showed that 5-HTT-/- mice exhibit significantly increased depression-related behavior compared to 5-HTT+/- and 5-HTT+/+ mice exclusively in response to repeated forced swimming, but not to a single exposure to the forced swim test. However, as the exaggerated floating behavior returned to baseline level during the first trial of the following days (day 2 and 3), and the fact that this increased immobility of 5-HTT-/- mice was unique to the more aversive WM test gives the idea that 5-HTT-/- mice are more sensitive to the aversive situation and show more despair during the second and third WM trial than their 5-HTT+/- and 5-HTT+/+ littermates instead of actively coping with the stressful situation. 

The article "5-HTT Deficiency Affects Neuroplasticity and Increases Stress Sensitivity Resulting in Altered Spatial Learning Performance in the Morris Water Maze but Not in the Barnes Maze" was published in 2013. Journal: PLoS One.

### Increased stress sensitivity of mice deficient for the 5-HTT may be responsible for their altered performance in the aversive WM

In contrast to the WM the BM does not utilize the fear of drowning as a strongly aversive stimulus, and therefore was already shown to result in lower blood plasma stress hormone levels [76]. Moreover, spatial learning was shown to be inversely correlated with corticosterone levels in the WM, but not in the BM, suggesting that performance in the WM may be more affected by test-induced stress [76]. The aversiveness of the WM is further substantiated by the fact that WM induces hypothermia as a 2 min swim in the WM is reported to decrease the core body temperature by 4.5°C [92]and five swims of 45 sec with a very short inter trial interval are reported to lead to a rectal temperature drop of 9°C [93]. It is well-known from other behavioral tasks that high levels of stress can influence the animal's performance [94]. In accordance with the study of Harrison and co-workers [76] we detected significantly increased corticosterone levels in WM-tested compared to BM-tested mice 15 min after the start of one single trial, but interestingly not in mice after the first trial on the second testing day. Although there was no significant gene by treatment interaction WM-tested 5-HTT deficient mice tend to exhibit higher corticosterone concentrations compared to mice of the same *5-HTT* genotype after BM experience in both stress hormone cohorts. Moreover, repeatedly experiencing any of the two spatial learning tests resulted in *5-HTT* genotype differences with highest plasma corticosterone levels in 5-HTT-/- mice, while 5-HTT+/+ mice seemed to habituate regarding their stress response. These *5-HTT* genotype differences are in accordance with former studies analyzing glucocorticoid and Adrenocorticotropic hormone (ACTH) levels in mice of different *5-HTT* genotypes in response to stressors such as handling and injection [95,96]. Furthermore, an exaggerated adrenalin/epinephrine release into plasma could be shown as a reaction to 15 min of immobilization [97], whereas tyrosine hydroxylase mRNA expression after this type of acute stress in 5-HTT+/+ and 5-HTT-/- mice was not changed. In line with most previous studies our 5-HTT-/-, 5-HTT+/- and 5-HTT+/+ mice exhibit similar basal glucocorticoid levels [34,98-100]. That is why the observed *5-HTT* genotype differences after repeated spatial learning test performance can be regarded as a result of gene by stress experience interaction and point to an altered stress sensitivity of 5-HTT deficient mice. Therefore, the assumed different levels of aversiveness of BM and WM in combination with an increased stress sensitivity of the tested 5-HTT deficient animals might explain inferior learning performance in the WM as an altered responsiveness of 5-HTT-/- mice towards a seemingly inescapable aversive WM environment without actually affecting spatial learning abilities *per se*. 

The article "5-HTT Deficiency Affects Neuroplasticity and Increases Stress Sensitivity Resulting in Altered Spatial Learning Performance in the Morris Water Maze but Not in the Barnes Maze" was published in 2013. Journal: PLoS One.

Comparable to the results of 5-HTT deficient mice or rats, human individuals carrying the S-allele of the *5-HTT* gene exhibit a greater reactivity to stress. This relation is supported by human imaging studies, which have found that carriers of the S-allele display greater amygdala activation in response to fearful stimuli [101], that is dependent on 5-HTT availability [102]. Moreover, stressful life events were shown to correlate with the severity and number of episodes of major depression in the individuals carrying lower expressing *5-HTT* genes [103,104]. 

### Increased number of IEG-positive cells in the hippocampus of 5-HTT-/- mice compared to 5-HTT+/+ littermates point to higher baseline hippocampal activity levels in mice with lifelong 5-HTT deficiency

We were aware that the chosen time-point was not ideal for IEG expression analysis related to effects of the exposure to the different test apparatuses as in immunocytochemistry as well as in mRNA-studies IEG protein/mRNA expression had been shown to peak within the first hours (protein) or even minutes (mRNA expression) after different learning tests or stress exposure and then return to baseline after a maximum of 24 hrs [51,105-107] . But, as the survival time of 60 hrs after 5 days of learning test exposure seems to be perfect for the analysis of early neurogenesis stages we decided to quantify the number of cFos- and Arc-positive cells in the DG of our mice (behavior-cohort) sacrificed 60 hrs after the last spatial learning test. This was done, as we aimed at testing the hypothesis suggested by [22] that 5-HTT-/- brains display a “stressed” morphological phenotype and hoped to find increased numbers of IEG-expressing cells in the hippocampus of 5-HTT-/- compared to 5-HTT+/+ mice. 

The article "5-HTT Deficiency Affects Neuroplasticity and Increases Stress Sensitivity Resulting in Altered Spatial Learning Performance in the Morris Water Maze but Not in the Barnes Maze" was published in 2013. Journal: PLoS One.

As expected, we did not detect differences between the number of Arc positive cells in mice of the different treatment groups (CONT, BM, WM), but overall *5-HTT* genotype effects with significantly higher number of Arc-ir cells in the DG of 5-HTT-/- mice compared to 5-HTT+/+ mice. In contrast to our results, significantly reduced Arc mRNA expression was detected in the whole hippocampus of 5-HTT deficient rats, irrespective of hippocampal subregions and different layers [108]. Additionally, Eriksson et al. found that Flinders sensitive line (FSL) rats display emotional memory impairments accompanied by reduced Arc mRNA expression specifically in brain regions implicated in cognitive processing such as the dentate gyrus [109]. These results, however, do not necessarily contradict our results, as our study analyzed the total number of Arc-ir cells and exclusively focused on the granule cell layer of the DG. The fact that both, the Molteni study using 5-HTT deficient rats and our study using 5-HTT deficient mice revealed *5-HTT* genotype dependent alterations in baseline Arc expression may be explained by a compensatory mechanism in response to the lifelong altered extracellular and intracellular 5-HT-levels, which could be the neurobiological correlate of heightened anxiety. This notion is supported by the fact that serotonergic signaling and Arc thus have opposing effects on AMPA type glutamate receptor (AMPAR)-trafficking. While serotonergic signaling enhances trans-synaptic signaling efficiency via the insertion of AMPARs into synapses at postsynaptic neurons [110], Arc expression is reciprocally regulated by activity and facilitates the endocytosis of certain AMPARs resulting in reduced AMPARs surface expression [111]. The latter possibly resulting in an increase of the threshold for LTP followed by altered learning and memory processes. From the results of our quantitative immunohistochemistry study we cannot tell if Arc is overexpressed in single cells of the DG in 5-HTT-/- compared to 5-HTT+/+ mice. However, one could speculate that having more cells expressing Arc at baseline coincides with the overexpression in single cells. 

Regarding cFos, significantly increased numbers of cFos-ir cells were found in the septal hippocampus of 5-HTT-/- compared to 5-HTT+/+ mice. From a number of older studies it is known that cFos is upregulated in the DG in response to various acute stressors including immobilization, noxious stimulation and hyper osmotic stress [65,112] as well as in response to chronic defeat [113]. Interestingly, chronic restraint stress has also been found to cause a significant increase in 5-HT [114]. This gives reason to assume that 5-HTT-/- mice, which have higher basal extracellular 5-HT levels and thus resemble chronically stressed mice, are closer to a “stress threshold” than 5-HTT+/+ mice. Beyond that, it is known that chronic restraint stress causes atrophy of apical dendrites in CA3 pyramidal neurons of the hippocampus [115-120] and that this atrophy is correlated with impaired spatial memory performance. Interestingly, the atrophy as well as the impairment could be reversed by lowering extracellular 5-HT pharmacologically in the septal hippocampus [121,122].

The article "5-HTT Deficiency Affects Neuroplasticity and Increases Stress Sensitivity Resulting in Altered Spatial Learning Performance in the Morris Water Maze but Not in the Barnes Maze" was published in 2013. Journal: PLoS One.

Finally, the increased baseline expression of the two IEGs Arc and cFos shown in this study may have promoted the pronounced stress sensitivity of 5-HTT-/- mice. Thus, elevated Arc and cFos protein levels could represent a “stressed” brain phenotype in consequence of lifelong 5-HTT deﬁciency, thereby presenting the neurobiological correlate of increased stress sensitivity and heightened anxiety of 5-HTT-/- animals. 

### Increased adult neurogenesis in the hippocampus of 5-HTT-/- mice compared to 5-HTT+/+ littermates indicates a compensatory mechanism for lifelong increased extracellular 5-HT levels

*5-HTT* genotype effects regarding proliferation (Ki67) and neurogenesis (NeuroD) comprise 5-HTT-/- mice displaying more immunoreactive cells than 5-HTT+/+ animals. This result is quite feasible when keeping in mind that, first, the lack of 5-HT clearance in these mice results in a persistent 5 to 13-fold increase of 5-HT concentrations in the extracellular space [16,17], and second, that 5-HT is a positive modulator of stem cell proliferation and neurogenesis in the adult hippocampus [123-125]. Schmitt et al. have already achieved similar results in 2007, albeit only in aged (14 months old), and not in young adult mice. More recently, immunoreactivity for the neurogenesis marker doublecortin was discovered to be increased in the dentate gyrus of 5-HTT-/- rats in comparison with 5-HTT+/+ rats [126]. In this study Schipper et al. were able to normalize both, increased anxiety-like behavior of 5-HTT-/- rats and altered neurogenesis level by feeding 5-HTT-/- animals a special diet. This led them conclude, that the behavioral effect of their special diet was probably conveyed via normalizing neurogenesis [126]. Thus, increased stem cell proliferation and neurogenesis in 5-HTT-/- animals can be discussed as neurobiological correlates to the increased anxiety-like behavior of 5-HTT-/- mice and rats.

Beyond the overall increased aN levels in 5-HTT deficient compared to 5-HTT+/+ mice our statistical tests revealed a significant gene by environment interaction of Ki67-ir cells in the SGZ of total DG. The number of Ki67-ir cells was shown to be different between naïve and WM-tested 5-HTT+/+ mice, with those tested in the WM displaying more proliferating cells in the SGZ than naïve animals. Moreover, naïve 5-HTT-/- mice already exhibited a trend towards higher numbers of proliferating cells compared to 5-HTT+/+ mice, whereas there was neither a significant difference between the two genotypes after BM or WM nor a significant effect of treatment within 5-HTT-/- mice. Considering that stress decreases aN [70,72,127,128], and that 5-HT increases aN [73], these lacking effects might be the result of the antagonistic effects of increased 5-HT-levels on the one hand, and the increased stress sensitivity of 5-HTT-/- mice on the other hand. 

The article "5-HTT Deficiency Affects Neuroplasticity and Increases Stress Sensitivity Resulting in Altered Spatial Learning Performance in the Morris Water Maze but Not in the Barnes Maze" was published in 2013. Journal: PLoS One.

There were two studies dealing with the impact of WM-testing on hippocampal aN in the rat, which resulted in contradictory outcomes. The first one, which is also probably the most well known study to convey the enhancing effects of spatial learning on aN, was carried out by Gould and colleagues in 1999 [74] In their experiment rats were exposed to 4 WM trials per day for 4 consecutive days with maximum trial duration of 60 s. The number of proliferating cells was increased in rats that had undergone hippocampus-dependent spatial learning in the WM compared to all control groups (including a swim-stress group)[74]. In the second study, Namestkova and co-workers [129] subjected rats to the same procedure, but for 15 consecutive days. This long-lasting treatment caused a significant decrease in progenitor cell proliferation in the granule cell layer of the hippocampus compared to controls [129]. In our study mice were subjected to WM training on 5 consecutive days and thus resembling the Gould et al. study more than the Namestkova et al. study. Therefore, the detected increase of proliferating cells in WM trained 5-HTT+/+ mice found in our study may be regarded as a result of spatial learning. 

The finding that there was no significant difference between the differently treated 5-HTT-/- mice, including the fact that there was already a trend towards higher numbers of proliferating cells in naïve 5-HTT-/- vs. 5-HTT+/+ mice suggests that this embodies a ceiling effect, that 5-HTT-/- mice are closer to a “stress threshold” than 5-HTT+/+ mice. A comparable ceiling effect was already described by Nietzer and co-workers, who found higher spinogenesis in the amygdala in naïve 5-HTT-/- vs. 5-HTT+/+ mice [22]. As stress-dependent effects were not detected in 5-HTT-/- animals, the authors concluded that these mice display a “stressed” morphological phenotype as a consequence of long-life 5-HTT deficiency per se [22]. We suggest that such ceiling effects act as a part of a compensatory mechanism, which probably sensitizes or desensitizes for future additional stress experience. Additionally, it may explain why spatial learning over a moderate time in the WM – normally a positive modulator of progenitor cell proliferation [74] – had no effect on proliferation in the SGZ of 5-HTT deficient mice. 

The article "5-HTT Deficiency Affects Neuroplasticity and Increases Stress Sensitivity Resulting in Altered Spatial Learning Performance in the Morris Water Maze but Not in the Barnes Maze" was published in 2013. Journal: PLoS One.

Regarding the number of NeuroD-ir cells, a positive correlation between the number of NeuroD-ir cells in 5-HTT-/- mice subjected to the WM and their overall performance (AuC) could be found revealing that mice with lower numbers of NeuroD-ir cells performed worse in the WM. The modulation of aN by WM test experience and the detected correlation between the number of newborn neurons and the learning performances point to an important role of this neuroplasticity phenomenon in the handling of stress and in learning and memory processes. This discovery is consistent with a study of human hippocampal neurogenesis by Coras and colleagues showing that patients with low numbers of proliferating progenitor cells and new-born neurons *in vivo* and *in vitro* showed a severe learning and memory impairments [130]. 

### Different hippocampal subregions with different connectivities and functions

Moser and Moser suggested that the hippocampus is functionally different along its septotemporal axis [131]. In rodents, spatial and episodic memory appears to depend on septal but not temporal hippocampus [64,132,133]. On the other hand, the temporal but not the septal hippocampus is thought to mediate stress responses and thus emotional behavior[134-137]. In rats it is well established that serotonergic neurons of the median raphe nucleus primarily project to the septal part of the hippocampal formation rather than in its temporal part [138]. Additionally, within the septal hippocampal formation median raphe neurons terminate throughout the rostrocaudal extent of the DG. Within the DG these projections are closely confined to the SGZ with more representations in the suprapyramidal blade than in the infrapyramidal blade of the DG [138]. Considering this, it is not surprising, that most significant *5-HTT* genotype effects regarding cell activation (Arc/ cFos) or neurogenesis (Ki67/ NeuroD) were found in the suprapyramidal blade of the DG. However, only environmental factors like spatial experience, transient forebrain ischemia, or kainic acid administration, have been found to cause region specific effects regarding IEG-expression, aN and or even morphological changes [139-143]. So far, this is the first study showing region-specific genotype differences in aN and the number of IEG expressing cells. 

In summary, our BM and WM results point to comparable spatial learning capabilities of mice with different *5-HTT* genotypes, but the performance differences of 5-HTT deficient mice in the WM task support a role for the 5-HTT in the hippocampally-mediated interaction between stress and spatial learning performance. Moreover, we suggest that increased IEG expression and aN levels observed in the hippocampus of 5-HTT deficient mice can be the neurobiological correlate of emotion circuit dysfunction and heightened anxiety as 5-HTT-/- animals *per se* display a “stressed” phenotype as a consequence of long-life 5-HTT deﬁciency. The experience of BM and WM tests results in either altered or even absent neuroadaptive increases in IEG and aN marker expression in 5-HTT-/- animals reducing adequate compensation processes and resulting in exaggerated behavioral responses e.g. in the more aversive WM. 
